# Validity and Reliability of Semiquantitative Food Frequency Questionnaires for Assessing Nutrient Intake among Preschool Children in Northwest China

**DOI:** 10.1155/2022/1677252

**Published:** 2022-01-12

**Authors:** Yonghong Ma, Jiao Tan, Zhijun Tan, Lei Shang

**Affiliations:** ^1^Department of Health Statistics, School of Public Health, Airforce Military Medical University, Xi'an 710032, Shaanxi, China; ^2^Department of Health Statistics and Epidemiology, School of Public Health, Xi'an Medical University, Xi'an 710021, Shaanxi, China; ^3^Research Center for Medical Prevention and Control of Public Safety of Shaanxi Province, Xi'an 710021, Shaanxi, China

## Abstract

**Background:**

Considering the lack of valid and reliable food frequency questionnaires (FFQs) for nutritional epidemiological studies in China, it is necessary to develop an effective one for assessing nutrient intake among preschool children. The aim of this study was to evaluate the validity and reliability of newly developed FFQs for assessing food and nutrient intakes among preschool children in Northwest China.

**Methods:**

Semiquantitative 67-item FFQs were developed and validated. In total, 326 children (aged 2–6 years) were recruited from three different cities in Northwest China. All subjects were asked to complete the FFQs twice with a six-month interval period for test-retest reliability. Apart from the FFQs, a 3-day food record (3-DFR) was also carried out to evaluate the validity of the FFQs.

**Results:**

There was no significant difference in the nutrient intakes of preschool children between the two FFQs (*P* > 0.05), and these two FFQs demonstrated a positive correlation (*P* < 0.05). Spearman's coefficient correlation values ranged from 0.222 (“Selenium”) to 0.832 (“Energy”). The intraclass correlation coefficient values ranged from 0.282 (“Selenium”) to 0.882 (“Energy”). With regards to the validity of FFQs, nutrient intakes from FFQs were greater than 3DR dietary recalls (*P* < 0.05). After adjusting for total energy and intraindividual variation, all nutrient intakes showed a positive correlation (*P* < 0.05), and these correlations became stronger. According to the quartiles of nutrient intakes, the exact agreement between the FFQs and 3DR dietary recalls ranged between 40% (“Selenium”) and 70% (“Energy”), and grossly misclassified was low (12.5%).

**Conclusions:**

The findings of this study indicate that the designed FFQs exhibit good test-retest reliability and moderate relative validity. Hence, the FFQs can serve as an important tool for the large-scale assessment of food and nutrient intakes among preschool children (in the mentioned areas of China).

## 1. Introduction

A healthy dietary pattern not only promotes the growth and development of children but also improves their health and well-being. There has been growing evidence to support the association between dietary patterns and the risk of chronic diseases in preschool children, such as diabetes, hypertension, cardiovascular disease, and so on [1]. Preschool children who are living in rural areas and whose parents are spending less on food usually consumed more vegetables and cereals but had limited intakes of aquatic products, meat, nuts, and dairy products [2]. On the contrary, those living in households with high food expenditures consumed more aquatic products, meat, nuts, and dairy products [2]. This contrast highlights the need for the accurate and reliable assessment of nutrient intake in preschool children so that instruments that seek to examine dietary patterns must be continuously evolved to meet the challenges.

Numerous methods have been established for the measurement of dietary intake; however, a simple and cost-effective technique is still lacking. The food frequency questionnaires (FFQs) have become increasingly popular for the estimation of dietary intake in large population groups. FFQs were preferred to 24-hour dietary recall (24-HDR) because of their high response rate and low respondent burden. Another reason is that FFQs can provide dietary information over a long period of time without changing common eating habits [3]. However, the limitation of FFQs lies in their capability to quantify the absolute intakes of specific foods or nutrients.

To date, more and more FFQs have been developed and validated for epidemiological studies in China [4–7]. However, most of them are specifically designed for the adult population, and thus, they may not be suitable for preschool children. Therefore, it is important to evaluate the reliability and validity of FFQs in the population of interest. Although several FFQs have been specifically designed for preschool children [8, 9], these FFQs may not be relevant to the contexts of preschool children in Northwest China. The purpose of this study was to examine the reliability and relative validity of semiquantitative 67-item FFQs for assessing food and nutrient intakes in preschool children.

## 2. Methods

### 2.1. Research Subjects

Preschool children aged 2–6 years were recruited from Xi'an, Xining, and Lanzhou cities (Northwest China). The specific location is shown in Figure 1 (the three cities were highlighted). Written informed consent was obtained from each child's parents or guardians before we started the questionnaire survey. Between March 2019 and October 2019, 400 participants were invited to answer the FFQs three times. The first FFQ (FFQ1) was conducted in person by a trained interviewer at the beginning and the second FFQ (FFQ2) 5 weeks later. The 3-day dietary record (3DR) was conducted one week after FFQ1. The inclusion criteria were as follows: (i) preschool children in Northwest China and (ii) no history of medical illness that may alter food intake. A total of 326 subjects were finally included for the analysis.

### 2.2. Study Design

The design of the study is shown in Figure 2. The questionnaire was gradually improved and compiled by our team on the basis of a comprehensive investigation on the diet habit of preschool children in China's Northwest region and on the basis of a thorough review of the relevant literature. After being investigated three times and modified, a formal semi-FFQ was formed. The formal FFQ was used to investigate 326 preschool children in Xi'an, Xining, and Lanzhou for the first time. One week later, a three-day diet review of the subject was conducted. In order to prevent the influence of the season on the diet, four weeks later, the third dietary survey was conducted to verify the results of the first questionnaire survey. In most cases, the children's parents are compliant with the arrangements administered by the kindergarten. Our research consequently utilized a stratified cluster sampling method to select the kindergartens across distinct districts. We recruited the preschool children's parents who voluntarily chose to participate in our project from every selected kindergarten as the subjects of our study.

### 2.3. Food Frequency Questionnaires

The semiquantitative FFQs were developed based on a review of the literature and previous FFQs established for the Chinese population [4, 10, 11]. The FFQs consisted of three major sections. The first section included personal questions related to age, gender, height, weight, and the levels of daily activities (i.e., the amount of time dedicated to physical exercise and sleep every day). The second section of the FFQs contained informative questions about the intake frequencies of 67 foods and beverages in the past month. The foods were classified into the following groups: cereals and cereal products, stuffing food, sweet food, deep-fried food, livestock meat, poultry meat, aquatic products, animal organs, milk and products, eggs and products, soy products, fruits, dark leafy vegetables, light leafy vegetables, mushroom vegetables, and beverages. Specific types of food are shown in Table 1. All participants were asked to indicate the frequency of their food ingestion by 9 response options ranging from “never” to “more than 3 times per day.” In the last section of the FFQs, a diagram of medium serving sizes was constructed according to the food's instruction manuals.

To calculate nutrient intake, the standard portion (in grams) was multiplied by the frequency of food intake. Each food item has a food-code linkage corresponding to the code number listed in the Chinese Food Composition Tables. The adjustment of nutrient losses during cooking was carried out, especially for dishes. The nutrient intakes for each participant were calculated using Food-Calc and Chinese Food Composition Tables [12, 13].

#### 2.3.1. -Day Food Record for Improvement and Validation

One time of 3-day food record (3-DFR) was used to estimate the seasonal and day-to-day variations in dietary habits [14]. For each 24-HDR, the participants' parents or caregivers were asked to recall their food consumption in the past day. The 3-day food record according to the design, at least one of three days, must be investigated on the children's diet during the weekend. The types and quantities of nutritious foods consumed were recorded in details. The collected dietary intake data (in gram or milliliter) were coded and examined by a dietitian prior to further analysis.

### 2.4. Statistical Analyses

All data were entered into Statistical Package for the Social Sciences 20.0 (SPSS 20.0) spreadsheet and checked by a trained nutritionist. The respective dietary intake for different types of food in our study was calculated based on the database named “Chinese Food Composition Inventory (6th Standardized Edition)” using the standardized nutrients calculator jointly developed by the Chinese CDC (Chinese Center for Disease Control) and the Institute of Nutrition and Food Safety, which are also the institutes that established the aforementioned food database. Dietary and nutrient intake results, along with demographic data, were analyzed using SPSS. Descriptive analysis was employed to compare the differences in basic characteristics (mean age, BMI, gender, residence area, and maternal education) among the research subjects. For the reliability test (FFQ 1 vs. FFQ 2), the intraclass correlation coefficients (ICCs) were determined, followed by Spearman's coefficient correlation (SCC) test. ICC is considered a suitable approach to evaluate the consensus between FFQs 1 and 2 as it can analyze between- and within-subject variabilities [15]. In addition, the nutritional variables were classified into the same or adjacent quartile (correctly classified, CC). Otherwise, they were classified into a nonadjacent quartile (grossly misclassified, GM). A *p* value of less than 0.05 was deemed statistically significant.

## 3. Results

The general characteristics of the 326 children who participated in this study are shown in Table 2. There was a uniform distribution of gender and age among the study participants. All subjects were from Xi'an, Lanzhou, and Xining cities. Most of the parents were highly educated, with a college degree, and the above accounted for 61.96%. Of the 326 participants, 11.04%, 9.20%, and 22.39% were measured to be underweight, overweight, and obese, respectively.

Table 3 shows the test-retest reliability of FFQs for preschool children. After the *t*-test of each nutritional variable in FFQ 1 and FFQ 2, the results showed that the most nutrient intakes of children were not significantly different between the two FFQs (*P* > 0.05). Vitamin C, sodium, selenium, and magnesium are statistically different between FFQ1 and FFQ2 (*P* < 0.05). The median of SCC for all nutritional variables in the test-retest reliability study was 0.511. The SCC values ranged from the lowest (*r* = 0.222) for “Selenium” to the highest (*r* = 0.832) for “Energy” (all *P* > 0.05). The median ICC was 0.546 (range: 0.282–0.882), and 63% (12 of 19) of the “Energy” and nutrients had ICC values of more than 0.5.

Table 4 demonstrates the relative validity of FFQs for preschool children. A_FFQ represents the median nutritional value of FFQ 1 and FFQ 2, and 3DR means the average of three days. After the paired *t*-test of each nutritional variable in A_FFQ and 3DR, the results showed that most of the nutrient intakes of the children were not significantly different between the two FFQs (*P* > 0.05). However, fat, vitamin E, iron, and selenium are statistically different between A_FFQ1 and 3DR (*P* < 0.05). Notably, the SCC values of more than 0.5 were observed for over 61% (11 of 19) of the “Energy” and nutrients in the FFQ. The median SCC was 0.531, and the individual SCC ranged from 0.168 (“Selenium”) to 0.70 (“Energy”). The median ICC was 0.521 (range: 0.210 to 0.825), and 53% (10 of 19) of the “Energy” and nutrients had ICC values of more than 0.5. Besides, the exact agreement between FFQ and 3DR was the highest (70%) for “Energy” but the lowest (40%) for “Selenium.” The mean percentages of CC and GM for all nutritional variables were 55.4% and 12.5%, respectively.

## 4. Discussion

In the present work, we evaluated the reliability and validity of FFQs developed for preschool children living in Northwest China. The test-retest reliability of FFQs was assessed by comparing the FFQs twice in the six-month interval period. At the same time, the relative validity of FFQs was determined against 3DR. The results demonstrated that our FFQs provided good quantitative estimate of nutrient intakes in healthy preschool children.

### 4.1. Test-Retest Reliability

FFQs displayed excellent test-retest reliability with the median ICC of 0.546 (range: 0.282 to 0.882), which is relatively similar to the range (0.37 to 0.96) reported in previous studies [16, 17]. However, the reliability of FFQs for preschool children is slightly lower than that for adolescents and adults [15, 18]. The reason may be that preschool children have greater dietary variation compared with adolescents and adults. Besides, an interval of more than half a year can result in an underestimation of FFQ retest reliability when compared to a shorter study interval [17, 19]. Cade and coworkers [20] have suggested that it is not wise to administer a questionnaire at a very short interval as respondents may remember their answers, while some changes in dietary patterns may be observed if the interval is too long.

### 4.2. Relative Validity

In this study, the estimate of energy and nutrient intakes was higher for FFQs than for 3DR, and also, it is higher compared to the results of other age groups of children [8, 10, 21]. The dietary survey of preschool children is answered by their parents or caregivers. They often have high expectations for their child's dietary intake, and the food provider may not be always the same for each meal of a child. This can lead to an overestimation of the child's daily food and nutrient intake.

By comparing the nutrient and energy intakes estimated from the FFQs with the reference method (3DR), a lack of exact consensus could be observed. The median of SCC between FFQs and 3DR was 0.545, varying from 0.168 to 0.814. SCC is a standard indicator for most validation studies, in which *r* < 0.49 indicates poor agreement and *r* > 0.5 indicates good agreement [20, 22]. In this study, twelve of the nutrients had a positive correlation coefficient (*r* > 0.5), while fifteen of the nutrients were over the threshold value (*r* > 0.4), which are quite consistent with findings from previous studies [20, 23].

Considering that 3DR can only measure short-term dietary intake, it is necessary to conduct multiple dietary surveys for each research subject to accurately estimate the dietary intake during the entire FFQ study period. However, such a large number of repeated measurements is difficult to be achieved in actual work, and it may cause a decrease in the number of subjects and changes in the behavior of the research subjects. Willett [24] found that the ICC method requires only a few repeated measurements (more than twice) on the survey subjects, and it can be used to obtain a reasonable estimate of the true value of the correlation coefficient. The median of ICC between FFQs and 3DR was 0.521, varying from 0.210 to 0.825, and these results are similar to those of foreign children and adolescents. ICC was used to reduce the influence of factors, such as measurement times, and a close to true correlation coefficient was obtained, revealing that the FFQs in this study exhibit good validity.

The proportion of subjects classified into one quartile (within the same or adjacent category) by FFQs and 3DR average was 55.3%. Extreme misclassification into the opposite quartile was 12.5% for all energy and nutrients. It was similar to the results of the FFQs study (<10%) compiled by Inge Huybrechts for Flemish preschoolers [25]. For the purpose of epidemiological research, the questionnaire has a good ability to distinguish the nutrient intake level of each research subject, which is more meaningful than obtaining the average intake.

Nevertheless, there are some limitations to the present study. One limitation is the relatively low response rate. The reason may be that the preschool child's parents have difficulty in understanding the information of average intake, food size, etc., and this research takes a long period of time. A low response rate of FFQs has also been reported in some validation studies [26]. During the course of data analysis, it has been discovered that 61.96% of the preschoolers' mothers who participated in our study had a college education, which demonstrates that their average education level is fairly high. Mother plays an important role in preschoolers' nurturing. It has been shown in relevant studies that the higher the mothers' education levels, the healthier the acquired dietary structure of their children and the fewer the types of unhealthy food consumed by them [27, 28]. Therefore, we believe that our study might have underestimated the quantity and the number of the types of unhealthy food consumed by preschoolers.

## 5. Conclusions

Although their effectiveness may be limited, the FFQs are developed based on the nutritional characteristics of a contemporary diet of preschool children and have been compared with similar related studies. In addition, the FFQs exhibit good test-retest reliability and moderate relative validity for assessing nutrient intake among preschool children in Northwest China. Furthermore, the high response rate and low respondent burden of the designed FFQs could make them more applicable for estimating nutrient intake in large-scale epidemiological studies.

## Figures and Tables

**Figure 1:** The location of the three research areas on the map of China (marked red).

**Figure 2:** The design of validity and reliability study of 326 preschool children in the north of China.

**Table 1:** Description of the food items included in the food categories and consumption rate of preschool children.

Food categories	Food name	Consumption times^a^	Consumption rate^b^ (%)
Cereals and cereal products	Rice, millet, black rice, noodles, steamed buns/cakes, rice porridge, etc.	533	98.52
Stuffing food	Stuffed bun, wonton/dumpling, etc.	312	57.67
Sweet food	Bread/cake/biscuits, etc.	387	71.53
Deep-fried food	Deep-fried dough sticks/oil cakes, etc.	256	47.32
Livestock meat	Pork/pork chops, beef, lamb, etc.	526	97.23
Poultry meat	Chicken, duck, goose meat, etc.	246	45.47
Aquatic products	Fish, shrimp, and other seafood.	209	38.63
Animal organs	Animal liver, animal blood clot, etc.	189	34.94
Milk and products	Milk, yogurt, soy milk, etc.	498	92.05
Eggs and products	Eggs, duck eggs, quail eggs, etc.	412	76.16
Soy products	Tofu, tofu shreds, dried tofu, soy milk, etc.	243	44.92
Pome fruits	Pome fruit such as apple/pear/papaya.	234	43.25
Stone fruit	Peach/plum/apricot/cherry and other stone fruits.	207	38.26
Berry fruits	Berry fruits such as grape/strawberry/pomegranate.	178	32.90
Citrus fruits	Orange/grapefruit and other citrus fruits.	161	29.76
Dark leafy vegetables	Spinach, lettuce, celery (stalks), rape, garland chrysanthemum, coriander, cabbage, and other dark vegetables.	478	88.35
Light leafy vegetables	Chinese cabbage, cauliflower, bean sprouts, and other light leafy vegetables.	268	49.54
Fruit vegetables	Potatoes, lotus roots, white radishes, cucumbers, garlic sprouts, tomatoes, eggplants, carrots, zucchini, and other vegetables.	218	40.30
Mushrooms and seaweeds	Mushroom, seaweed, black fungus, etc.	226	45.29
Beverages	Carbonated drinks, fruit juices, and other sugary drinks.	213	43.81

a: consumption times mean the respective consumption times of every single type of nutrient for every child within a month, and b: consumption rate means the total consumption ratio of the food in all survey subjects.

**Table 2:** Basic characteristics of the study participants.

Characteristics		Subjects	Percentage
Gender	Male	167	51.23
	Female	159	48.77
Age	3-4 years	137	42.02
	4-5 years	115	35.28
	5-6 years	74	22.70
Residence area	Xi'an	196	60.12
	Lanzhou	69	21.17
	Xining	61	18.71
Maternal education	Junior and below	36	11.04
	Senior	88	26.99
	College and above	202	61.96
BMI	Underweight	36	11.04
	Normal	187	57.36
	Overweight	30	9.20
	Obesity	73	22.39

**Table 3:** Test-retest reliability of FFQs for preschool children.

Item (units/d)	FFQ 1		FFQ 2		*P* value	SCC	ICC	%difference
	Median	(P25–P75)	Median	(P25–P75)				
Energy (kcal)	1669.69	(1337.62, 1951.31)	1935.73	(1542.00, 2167.31)	0.063	0.832	0.882	15.9
Carbohydrates (g)	215.49	(170.90, 255.88)	243.09	(195.28, 287.05)	0.231	0.599	0.669	12.9
Protein (g)	70.00	(55.19, 86.85)	79.02	(62.17, 92.15)	0.506	0.615	0.688	13.1
Fat (g)	48.87	(39.29, 63.87)	55.75	(40.16, 73.56)	0.162	0.622	0.613	14.5
Dietary fibre (g)	19.00	(14.68, 25.60)	22.09	(17.10, 28.04)	0.245	0.528	0.607	16.9
Cholesterol (mg)	365.08	(243.34, 468.42)	362.61	(243.34, 498.81)	0.304	0.547	0.553	-0.7
Vitamin A (IU)^*∗*^	993.54	(708.51, 1353.43)	1074.51	(823.16, 1493.34)	0.426	0.434	0.462	8.6
Thiamin (mg)	0.90	(0.67, 1.05)	0.94	(0.74, 1.13)	0.168	0.623	0.611	4.8
Riboflavin (mg)	1.39	(1.18, 1.74)	1.50	(1.23, 1.92)	0.242	0.561	0.551	8.5
Vitamin C (mg)	78.82	(52.41, 117.47)	94.57	(67.56, 127.50)	0.043	0.349	0.343	21.8
Vitamin E (mg)	13.95	(10.42, 20.33)	15.36	(11.85, 21.24)	0.089	0.493	0.483	11.1
Niacin (mg)	16.46	(12.92, 20.55)	18.11	(14.82, 22.89)	0.423	0.410	0.432	11.1
Calcium (mg)	641.20	(501.39, 808.48)	677.51	(549.22, 880.49)	0.476	0.551	0.436	6.3
Iron (mg)	25.29	(19.75, 34.55)	28.81	(22.57, 36.71)	0.135	0.556	0.521	15.7
Zinc (mg)	6.10	(4.70, 7.87)	6.92	(5.30, 8.52)	0.431	0.440	0.429	15.3
Phosphorus (mg)	886.31	(725.71, 1106.63)	942.74	(754.89, 1211.73)	0.542	0.589	0.508	7.3
Sodium (mg)	597.48	(492.03, 738.04)	694.44	(521.91, 866.27)	0.038	0.631	0.675	18.8
Selenium (mg)	19.31	(14.36, 28.57)	23.90	(15.52, 32.13)	0.046	0.222	0.282	27.8
Magnesium (mg)	372.18	(301.82, 515.16)	452.32	(349.58, 589.40)	0.025	0.528	0.546	25.4

*P* value of *t* test between FFQ1 and FFQ2. SCC: Spearman's correlation coefficient; ICC: intraclass correlation coefficient; %CC: the percentage of correctly classified; %GM: the percentage of grossly misclassified; %difference in nutrient intakes between FFQ 1 and FFQ 2; %difference = (FFQ 2 − FFQ 1/FFQ 1)  ^*∗*^ 100%.

**Table 4:** Relative validity of FFQs for preschool children.

Item (units/d)	A_FFQ		3DR		*P* value	SCC	ICC	%CC	%GM	%difference
	Median	(P25–P75)	Median	(P25–P75)						
Energy (kcal)	1802.71	(1439.81, 2059.31)	1522.51	(1313.65, 1704.75)	0.065	0.814	0.825	70	5	18.4
Carbohydrates (g)	231.44	(185.06, 273.14)	194.05	(162.54, 229.23)	0.058	0.703	0.671	65	9	19.3
Protein (g)	76.40	(61.74, 88.86)	66.94	(56.23, 77.21)	0.126	0.745	0.705	66	8	14.1
Fat (g)	55.09	(40.94, 66.53)	44.56	(36.97, 57.32)	0.047	0.545	0.707	59	15	23.6
Dietary fibre (g)	20.52	(16.03, 27.03)	17.97	(13.67, 23.12)	0.109	0.441	0.539	57	16	14.2
Cholesterol (mg)	378.93	(261.09, 482.60)	330.45	(223.63, 470.06)	0.164	0.310	0.313	48	17	14.7
Vitamin A (IU)^*∗*^	1057.42	(815.14, 1424.37)	998.99	(713.66, 1263.93)	0.336	0.306	0.306	44	18	5.8
Thiamin (mg)	0.90	(0.76, 1.09)	0.80	(0.66, 0.93)	0.368	0.707	0.649	56	9	12.5
Riboflavin (mg)	1.46	(1.22, 1.81)	1.37	(1.09, 1.63)	0.406	0.630	0.393	54	11	6.6
Vitamin C (mg)	87.26	(66.76, 121.74)	75.13	(48.81, 107.39)	0.132	0.321	0.338	45	17	16.1
Vitamin E (mg)	15.83	(11.57, 19.88)	12.73	(10.31, 17.46)	0.031	0.038	0.598	55	15	24.4
Niacin (mg)	18.24	(14.09, 21.58)	15.90	(13.23, 19.34)	0.147	0.554	0.397	50	9	14.7
Calcium (mg)	670.08	(527.28, 834.41)	638.63	(457.12, 800.97)	0.432	0.472	0.461	55	14	4.9
Iron (mg)	28.03	(21.33, 36.05)	23.67	(19.19, 33.02)	0.042	0.518	0.454	57	12	18.4
Zinc (mg)	6.72	(5.31, 8.02)	5.90	(4.88, 7.40)	0.165	0.411	0.350	49	18	13.9
Phosphorus (mg)	955.28	(744.88, 1097.16)	887.33	(695.83, 1056.06)	0.208	0.531	0.521	50	14	7.7
Sodium (mg)	649.36	(513.53, 809.68)	570.61	(473.25, 691.78)	0.252	0.664	0.721	68	5	13.8
Selenium (mg)	23.25	(15.81, 29.45)	18.55	(14.41, 28.86)	0.046	0.168	0.210	40	19	25.3
Magnesium (mg)	429.47	(336.37, 543.28)	369.20	(298.78, 488.18)	0.182	0.612	0.627	64	7	16.3

*P* value of *t* test between A_FFQ and 3DR. ICC: intraclass correlation coefficient; SCC: Spearman's correlation coefficient; %CC: the percentage of correctly classified; %GM: the percentage of grossly misclassified; %difference in nutrient intakes between A_ FFQ and 3DR; %difference = (A_FFQ − 3DR/3DR) × 100%.

## Data Availability

Data sharing is not applicable for this article.
